# Subgroup State Prediction under Different Noise Levels Using MODWT and XGBoost

**DOI:** 10.1155/2023/6406275

**Published:** 2023-01-31

**Authors:** Xin Zhao, Xiaokai Nie

**Affiliations:** ^1^School of Mathematics, Southeast University, Nanjing 211189, China; ^2^School of Automation, Southeast University, Nanjing 210096, China; ^3^Key Laboratory of Measurement and Control of Complex Systems of Engineering, Ministry of Education, Southeast University, Nanjing 210096, China; ^4^Shenzhen Research Institute, Southeast University, Shenzhen 518057, China

## Abstract

In medical states prediction, the observations of different individuals are generally assumed to follow an identical distribution, whereas precision medicine has a rigorous requirement for accurate subgroup analysis. In this research, an aggregated method is proposed by means of combining the results generated from different subgroup models and is compared with the original method for different denoising levels as well as the prediction gaps. The results using real data demonstrate the effectiveness of the aggregated method exhibiting superior performance such as 0.95 in AUC, 0.87 in F1, and 0.82 in sensitivity, particularly for the denoising level that is set to be 2. With respect to the variable importance, it is shown that some variables such as heart rate and lactate arterial become more important when the denoising level increases.

## 1. Introduction

Precision medicine has the sophisticated requirements for the accuracy and time efficiency of medical treatment that needs to make use of the physiological signals observed from the patients. The observation and analysis of these signals take a critical role in satisfying the treatment demand [1]. Usually, the clinical physiological signals are directly monitored and assessed by the clinicians in real time, such that patients' physical conditions can be grasped, and subsequently, the corresponding appropriate treatment is prepared and then implemented, including medicine usage and physical therapy. In particular, patients in severe situations may require uninterrupted on-site monitoring of clinicians to manage any possible emergent circumstance timely. For example, the intensive care unit (ICU) is a dedicated medical function for real-time monitoring of critically ill patients. Long-term and continuous commitment to medical care is challenging for the clinicians due to the demand on the high concentration on the treatment, which may inevitably cause fatigue and a negative impact on the performing efficiency, thereby likely incurring the unexpected medical accidents and medical costs, such that the favourable survival rate of the patients becomes difficult to be guaranteed. Therefore, a reliable monitoring scheme for the treatment is fundamental to achieve the precision medicine, as well as high-quality medical care [2].

Machine learning-based prediction of patients' state is a promising solution to elevating the performance of real-time monitoring for medical care, and considerably relieving the pressure arising from the instantaneous treatment following the situation observation [3, 4]. The framework of such state prediction allows patients to receive timely treatment by predicting patients' state prior to the state variation coming up, based on the past and currently recorded signal data, and assist clinicians to take necessary and associated actions to tackle the oncoming circumstance. This can largely lift the reliability of real-time medical care by means of providing the prediction for the clinicians in the form of observed variable value, emergent level, and trend of patients' physical conditions. In the practical situation, even a short period of time of prediction can be precious for clinicians and patients, which can reduce the tenseness of clinicians and largely improve the possibility of patients' survival in the intensive care.

Due to the complicated pathology, it is typically difficult to recognize a suitable model to accurately describe the features of the observed data. Statistical modeling, as a probabilistic way of describing the uncertainty phenomenon, aims to learn and analyze the underlying process that governs the generation of the data, and make predictions for the oncoming status [5]. For medical monitoring, the patient's physical condition is normally represented by different states, and each state indicates the associated level of severeness. Different from the general prediction from time series, states categorized in the healthcare system shows the class-imbalance phenomenon, that is, some state accounts for a large proportion of the whole observations, while some other state has a very small proportion of data. For example, among the available observations of the patient's state in the ICU, a frequently encountered case is that the state of being in danger which implies the patient's condition in emergent situation has a very low proportion of observations. In contrast, the majority of the observations are classified as the state of being relatively safe. Therefore, this leads to the apparent imbalance of probability distribution of the different states. Solving such issues is intractable by directly using the traditional simple machine learning approaches. There is one way to improve the prediction performance by reducing the weights of observations that are accurately predicted and increasing the weight of the incorrectly predicted observations. In this way, the impact of the observations with low proportions on the prediction results is expanded to reflect the underlying correlated relationship. Furthermore, the other challenge is that the established model is desired to have good interpretability, which is especially important for prediction-based medical assistance and can show the importance of the explanatory variables. In this context, based on the known properties of the physiological signal observations, the appropriate statistical model forms the basis of understanding the causality between the concerned variables and the generated data, and the modeling method is developed to characterize the state predicted using the available data.

To realize precision medicine, the interpretable models used for predicting patients' state requires the applicability of models to the patients with specific characteristics, therefore it is quite challenging to design a particular prediction model for a confined group of patients rather than the whole patients [6, 7]. The targeted patients having similar physical properties are applied with the same model, such that it is essential to understand how to group the patients based on their physical properties. In general, models are built for describing patients' physical conditions by ignoring the individual difference, and then cannot reflect the particularity; hence, such models lack the desired accuracy of predicting the state that is induced by the individual difference. To this end, the subgroups of the patients are determined before the modeling process. For each subgroup, the corresponding model may show better performance than the generalized model for the whole patient in terms of predicting the states associated with special observations. Such states are preferred to be predicted using the subgroup model instead of the generalized model established based on the whole observations. Another challenge of modeling comes from the random noise involved in the measured signals and caused by the monitoring devices or the measurement process. Leaving out the noise can decrease its impact on the original signals, and help improve the model performance. However, if the useful information contained in the signals is mistakenly treated as the noise, the model performance is then impaired, which is absolutely undesired. Therefore, determining the subgroup of patients and denoising the measured signals are imperative to obtain the effective prediction of the patient's state.

The highlights of this research include the following: (1) the wavelet transform method is adopted to leave out the noise contained in the measured physiological signals on different resolution levels, (2) the model XGBoost is applied to explore the relationship between the input signals and the response variable state, which has both good model performance and interpretability, and (3) a subgroup analysis is conducted before the modeling process. For each subgroup, a corresponding model is established, and the prediction process is conducted with its corresponding models.

In this article, a subgroup state prediction method based on wavelet transform is developed to deal with the noise involved in the measured physiological signals. The rest of the article is organized as follows: in Section 2, a review of the related literature is given. In Section 3, a systematic approach based on the model XGBoost and subgroup analysis are proposed in this research. In Section 4, the analysis of the real data using the proposed scheme is introduced. Concluding remarks and perspectives on the further research are given in Section 5. All the computations in this research were conducted using *R* [8].

## 2. Literature Review

Different from the conventional time series prediction in terms of data structure, longitudinal data or panel data prediction aims to address the issues of perspective data estimation for multiple dimensional datasets, which has the extensive applications in healthcare [9] and biological systems [10].

Logistic regression is a representative approach to state forecasting by handling categorical response variable. Logistic regression aims to estimate the probability of some event occurring by formulating the logarithm of the odds for the event in the form of a linear combination of independent variables. In [11] logistic regression models were used in genomic studies to analyze the genetic data linked to electronic health records, and their performance in the presence of positive errors in event time was evaluated. Castilla and Chocano [12] developed robust estimators and Wald-type tests for the multinomial logistic regression based on *ϕ*-divergence measures and analyzed the robustness of the approach. Dumitrescu et al. [13] proposed a credit-scoring model based on an adaptive LASSO logistic regression model with predictors extracted from decision trees, which give rise to a significant reduction in misclassification costs compared to the benchmark logistic regression. Leong et al. [14] studied a logistic regression approach to solving the field estimation problem using binary measurements. Schuster et al. [15] applied logistic regression to determine the presence of confounding bias in epidemiological research. Wang et al. [16] studied the sparsity-constrained logistic regression using the Newton method and showed the low computational complexity as well as the global and quadratic convergence properties of the proposed scheme. Ruiz et al. [17] applied the logistic regression model to analyze the risk factors associated with mortality in HIV patients admitted to ICU. The logistic regression has good performance in these applications but the limit is also obvious. As regression models are based on the assumption that observations are mutually independent and identically distributed, models based on parameter estimation are no longer suitable.

Nonparametric modeling approaches, including some typical machine learning methods [18, 19], are widely used to solve the medical state prediction issues. Gao et al. [20] utilized five machine learning models including logistic regression, random forest, LightGBM, XGBoost, and their ensemble model to early predict the occurrence of acute kidney injury (AKI) in the next 24, 48, and 72 h for ICU patients. Results show that their proposed gradient-boosting decision tree algorithms achieved relatively better performance than others. Greco et al. [21] applied logistic regression, balanced logistic regression, and random forest to predict mortality for COVID patients in emergency phases. Kurtz et al. [22] presented a structured data-driven methodology to construct the prediction models of the length of stay and 30 day mortality and compared the prediction performance by applying multiple classification methods to the ICU dataset. Ibrahim et al. [23] developed a scalable and robust machine learning framework to automatically predict adversity represented by mortality and ICU admission and readmission from time series of vital signs and laboratory results obtained within the first 24 hours of hospital admission. The solution comprises an unsupervised LSTM autoencoder for learning the optimal representation of the time series and a gradient-boosting model for refine prediction by incorporating static features. Lee et al. [24] developed a multiscale interval pattern-aware network to improve the temporal mining task based on electronic health. In general, such methods can have high accuracy of prediction but their interpretability may not be enough to support the medical decision if decision rules are required due to the complex structures of the models.

In addition to the aforementioned machine learning approaches, the ensemble method has become an attractive solution to achieving better performance. Wang et al. [25] introduced a weight decay random forest model to achieve ICU readmission classification based on sparse data and integrated the missing value analysis and the likelihood ratio test for the distribution characteristics of time series indicators. Munera et al. [26] applied a random forest model to predict the probability of ICU admission or hospital mortality, which was combined with a logistic regression model designed to select the clinical variables and laboratory results that best predicted the outcomes. Varghese et al. [27] employed the AdaBoost classifier to achieve early identification of COVID-19 patients at risk of a poor prognosis as defined by the need for ICU and mechanical ventilation, and showed the favourable performance of the AdaBoost classifier in the prediction. Wang et al. [28] proposed the model XGBoost to achieve timely and accurate prediction of the death probability of ICU patients. The results showed that XGBoost achieved obviously better performance than the traditional scoring methods. Based on the analysis above, the model XGBoost is suggested in this article.

The input variables are mainly the monitoring signals. The noise involved in the signals may influence the model performance. In order to explore how the level of noise influences the model performance, the denoising method should be applied before the modeling process. One of the methods is Fourier transform [29]; Zhai [30] used the fractional Fourier transformation for seismic data denoising. However, due to the disadvantages of Fourier transform, the wavelet transform is proposed in this article. The model maximal overlap discrete wavelet transform (MODWT) is a recently developed method in DWT, which can decompose the original time series into different resolution levels in a study [31]. The noise of high-resolution level can be removed afterwards. In addition to the denoising, the subgroup analysis should also be applied before the modeling process. The existng research normally assumes the data originates from one distribution, which does not vary across different individuals who have different baseline information. But the reality is that the model performance may differ across different individuals, as the data of different individuals differ. In this context, the paper proposes to use the decision tree model to divide the original data into different subgroups before other steps.

## 3. Methods

The baseline variables for analysis include age, sex, weight, and height. A decision tree model CART is applied to explore the relationship between each baseline variable and the dependent variable *Y* across all the patients. The subgroups can be determined accordingly, such as a group age < 38. For the subgroup *s*, *s* = 1,2, ⋯, *S*, the dependent data *Y*^*s*^ of patient *n* can be expressed as

(1) $$\begin{array}{c} Y_{n,\cdot }^{s}={\left[y_{n,1}^{s},y_{n,2}^{s},\cdots ,y_{n,T_{n}}^{s}\right]}^{T}\text{,} \end{array}$$

where *n* = 1,2, ⋯, *N* and *t* = 1,2, ⋯, *T*_*n*_. Generally, *y*_*n*,*t*_^*s*^ is a categorical random variable with a status value such as 0 or 1. The method developed by combing the results from different subgroups is called aggregated method in this research, while the method using all the data is referred to as the original method.

In order to explore how the level of noise influences the model performance, the explanatory variable *X*^*s*^ = [*X*_*n*,*k*,*t*_^*s*^] in group *s* is transformed with wavelet by using MODWT on resolution levels *j* as follows

(2) $$\begin{array}{c} W_{n,k,\cdot }^{s}=\left[\begin{array}{cccc} W_{n,k,1}^{s_{j}} & W_{n,k,2}^{s_{j}} & \cdots & W_{n,k,T_{n}}^{s_{j}} \end{array}\right]\text{,} \end{array}$$

where individual *n* = 1,2, ⋯, *N*, variable *k* = 1,2, ⋯, *K*, and time *t* = 1,2, ⋯, *T*_*n*_. The chosen wavelet basis is the Haar wavelet, which is defined as

(3) $$\begin{array}{c} \phi \left(t\right)=\left\{\begin{array}{cc} 1\text{,} & t\in \left[0,1\right)\text{;}\\ 0\text{,} & else\text{.} \end{array}\right. \end{array}$$

Using dilation and translation, the scaling function at resolution level *j* and location *r* is given by

(4) $$\begin{array}{c} \phi_{j,r}\left(t\right)=2^{j/2}\phi \left(2^{j}t-r\right)\text{.} \end{array}$$

Then, the scaling coefficients can be given by

(5) $$\begin{array}{c} W_{n,k,t}^{s_{j}}=<X_{n,k,t}^{s},\phi_{j,k}>\text{.} \end{array}$$

The higher resolution level implies that less noise is involved in the resultant scaling coefficients. For example, the variable on resolution level 0 is the original variable without denoising, while that on a higher level contains less noise and less detailed information. In order to achieve a robust model for each subgroup *s* at resolution level *k*, the data of all patients are combined into one data as follows

(6) $$\begin{array}{c} W_{k}^{s}={\left[W_{1,1:K,1:T_{1}-g}^{T},W_{2,1:K,1:T_{2}-g}^{T},\cdots ,W_{N,1:K,1:T_{N}-g}^{T}\right]}^{T}, \end{array}$$

where *W*^*s*^ is the explanatory variable for subgroup *s* across all the patients from 1 to *K*, and across all the possible observations from 1 to time *T*_*n*_ − *g* with *g* as the time gap. In this way, the corresponding *Y*^*s*^ is given by

(7) $$\begin{array}{c} Y^{s}={\left[Y_{1,g+1:T_{1}}^{s},Y_{2,g+1:T_{2}}^{s},\cdots ,Y_{N,g+1:T_{N}}^{s}\right]}^{T}\text{.} \end{array}$$

The model in use is the ensemble method XGBoost, which is short for eXtreme Gradient Boosting. As an additive model, it works by approximating its optimization function with the second order Taylor expansion. It fits the residuals generated from the last basic model and combines all the previous models to yield the final ensemble model.

(8) $$\begin{array}{c} P\left({\hat{Y}}^{s}=1\right)=XGBoost\left(W_{k}^{s}\right)\text{.} \end{array}$$

With a time gap *g*, at resolution level *j*, the model can be trained as *XG*Boost_*g*,*j*,*s*_ for subgroup *s*. Since one patient has four different baseline variables, the patient may belong to multiple subgroups such as age < 38 and height < 173. The predicted $P\left(\hat{Y}=1\right)$ for patient *n* is the averaged probability from those subgroups. For a new observation *X*_*n*,.,*t*_, to predict the dependent variable at time *t* with gap *g* at resolution level *j*, the prediction result is expressed as

(9) $$\begin{array}{c} P\left(\hat{Y}=1\right)=\frac{1}{m}\overset{m}{\underset{s=1}{\sum }}XGBoost^{s}\left(W_{k}^{s}\right)\text{.} \end{array}$$

By assuming $\hat{Y}=1$ if $P\left(\hat{Y}=1\right)>0.5$, the performance of the model is measured by the metrics AUC, F1, and sensitivity. Sensitivity and specificity are two metrics measuring the percentage of true positive (negative) observations out of the total positive (negative) observations. F1 and AUC are two metrics combining the information of sensitivity and specificity with higher values indicating the better performance of the model.

## 4. Real Data Analysis

This dataset was collected during routine care at the Department of Intensive Care Medicine of the Bern University Hospital, Bern, Switzerland [32]. It was designed to study the early prediction of circulatory failure in the intensive care unit. The dataset was collected during 2008 to 2016, including deidentified demographic information, physiological variables, diagnostic test results, and treatment parameters. The data have been preprocessed by Hyland et al. [33], and the imputed data to be analyzed in this research contain the 18 most predictive meta-variables with a five-minute time grid. The number of individuals is 33,905 whose observations range from hundreds to thousands. For more detail, please refer to Hyland et al. [33].

In order to explore how the baseline information influences the patient states, a tree model is built by using each baseline variable as the input and the percentage of the state value of one for each patient as the response variable. To build an adequate and small tree, the parameters of the tree are set to be 0.0001 for the complexity and 2 for the max depth. The results are shown in Figure 1. Although the chosen splitting criteria may not be significant under the hypothesis, it truly gives a reference for the subgroup analysis. By using the splitting criteria shown in Figure 1, the subgroup can be arranged as follows: (1) age < 38, (2) 38 ≤ age < 53, (3) 53 ≤ age < 68, (4) 68 ≤ age, (5) height <173, (6) 173 ≤ height < 183, (7) 183 ≤ height < 188, (8) 188 ≤ height, (9) sex = M, (10) sex = F, (11) weight < 63, (12) 63 ≤ weight < 93, and (13) 93 ≤ weight. In the rest of the analysis, the model is trained and validated under each subgroup. In this way, there are 13 different models. In order to compare the subgroup performance and the performance with all the observation without any subgroup, the model is further trained across all the individuals as the 14th model. In total, there are 14 models.

The model performance difference under the aggregated subgroup method or the original method has been explored under different noise levels 1,2,…, 8, and different prediction length gaps 1, 5, 10, and 20. The results in Figure 2 show that resolution level 2 is the best level among all the 8 choices, as it leaves out adequate noise but keeps the useful information. And thus, MODWT on resolution level 2 is proposed in the further research. In terms of the prediction gaps, the model XGBoost is robust under different gaps among all the performance metrics: AUC, F1, and sensitivity. Compared with the original method, the aggregated method shows better performance in most cases, with even 0.05 higher in the metric values sometimes.

From the results shown in Figure 3, the variable importance is measured by the percentage of being selected in the ensemble tree model XGBoost. The higher the percentage of the frequency, the more important the variable is. The first column of the figure shows the most important six variables, the second column shows the second important six variables, and the last column shows the least important variables. Across different denoising levels, variables show different behaviors. For example, in the second column, the variable heart rate becomes more important when the denoising level increases. The variable lactate arterial also becomes more important as well. The model performance shows little difference among different prediction gaps.

## 5. Conclusion

In this research, an aggregated method is developed by combining the results from the subgroup models trained by each subgroup data. The performance of this method is compared with the original method which has all the data trained in one single XGBoost model. The aggregated method generally has the better performance measured by AUC, F1, and sensitivity. The difference becomes obvious when the denoising level increases. The best noise level chosen is level 2, which can leave out redundant noise but still keep the useful information. When the denoising level increases from level 2, the model performance decreases obviously. When the prediction gap increases, the model performance is still robust. In terms of the variables involved, their performance is measured by their frequency to be chosen in the XGBoost model. The performance is compared under different denoising levels and prediction gaps. Results show that some variables such as heart rate and lactate arterial become more important when the denoising level increases.

With respect to the future research, the subgroup can be developed based on multiple variables instead of a single variable with one dimension. In addition to the four baseline information variables, more possible variables could be included for a better decision, for example, patient history. The model XGBoost can be further developed for a better performance with more interpretable variable importance.

## Figures and Tables

**Figure 1:** The decision tree result of how the baseline information influences the state's rate. The model in use is CART, and the baseline variables include age, height, sex, and weight. The state ratio for each individual is the percentage of state one over all his or her observations.

**Figure 2:** The results of the method under different noise levels and prediction gaps. The performance of the aggregated method based on 13 models is better than the method based on the original data without a subgroup.

**Figure 3:** The results of the variable importance. The frequency value is the percentage of one specific variable being selected in the ensemble XGBoost trees.

## Data Availability

The source code in the method is available from the corresponding author upon request. The real data in the application can be requested from Hyland et al. [33].
